# Treatment with Antiviral Drugs Will Significantly Inhibit the HIV-1 RNA POL Gene Expression and Viral Load in AIDS Patients

This article has been retracted.

**DOI:** 10.1155/2023/9910542

**Published:** 2023-04-14

**Authors:** Penghui Shi, Xiaodong Wang, Miaomiao Su, Juan Meng, Hao Wang, Weiguang Fan

**Affiliations:** ^1^Department of Laboratory Medicine, Baoding People's Hospital, Baoding City, Hebei Province 071000, China; ^2^Baoding People's Hospital, Baoding City, Hebei Province 071000, China; ^3^Department of Infectious Diseases, Baoding People's Hospital, Baoding City, Hebei Province 071000, China

## Abstract

**Objective:**

This study is to investigate the difference in HIV-1 RNA pol gene expression in AIDS patients before and after antiviral treatment and its effect on the expression level of CD4^+^/CD8^+^ T cells in peripheral blood.

**Methods:**

The participants included 200 AIDS patients who had undergone antiviral medication, and the quantity of HIV-1 RNA pol gene was determined using nested polymerase chain reaction (nPCR). The levels of CD3+, CD4+, and CD8+ T lymphocytes in peripheral blood were measured by flow cytometry before and after therapy. The receiver operating characteristics (ROC) curve was used to assess the impact of HIV-1 RNA pol gene expression and the CD4+/CD8+ ratio on the prognosis of AIDS patients.

**Results:**

After three months of therapy, the levels of HIV-1 RNA and viral load in the patients showed a drastic decline, while the levels of CD4+/CD8+ were markedly elevated (*P* < 0.05). Logistic analysis revealed that patients' viral loads were positively correlated with HIV-1 RNA and negatively correlated with CD4+/CD8+ (*P* < 0.05). The alanine aminotransferase (ALT), white blood cell (WBC) count, Serum creatinine (Cr), total cholesterol (TC), triglyceride (TG), and platelet (PLT) levels significantly increased following a 24-month therapy, while no significant changes were observed in the level of aspartate aminotransferase (AST), red blood cell (RBC), and neutrophil (NEU) (%). (*P* > 0.05).

**Conclusion:**

Antiviral drugs significantly inhibit the HIV-1 RNA POL gene expression and viral load in AIDS patients but upregulate the expression level of CD4^+^/CD8^+^ T cells in peripheral blood.

## 1. Introduction

AIDS is a systemic disease caused by the HIV virus infection [1]. It is characterized by high infectability for both men and women. According to reports, approximately 40 million people were afflicted worldwide in 2019, with 900,000 cases diagnosed in China. It is also reported that 30 to 40 thousand patients die of AIDS each year [2, 3]. No obvious symptoms can be found during the latent period of HIV infection; however, with the disease progression, symptoms such as fever, diarrhea, and significant loss of body weight may occur [4].

Currently, antiviral therapy is a major approach to AIDS management. Combination antiretroviral treatment (cART) has reduced HIV from a potentially fatal illness to a manageable infection. The current regimen consists of two or three antiretroviral medicines. Several antiretroviral medication classes have been created and classified based on their mechanism of action in the blockage of the HIV replication cycle [5]. In general, the different drug classes are (1) nucleoside and nonnucleoside reverse transcriptase inhibitors (NRTIs and NNRTIs), (2) protease inhibitors (PI), (3) fusion inhibitors, (4) entry inhibitors, and (5) integrase inhibitors (INIs) [6]. Monotherapy quickly leads to the emergence of resistant strains and treatment failure due to the high mutation rate of the HIV genome during viral replication. Inhibition of many different enzymes and blocking of important host-virus interactions during the virus life cycle are the key to completely blocking viral replication and preventing the development of drug resistance [7].

The research work on the treatment of AIDS by traditional Chinese medicine (TCM) can be traced back to the 1980s. Studies have confirmed that TCM has significant effects in regulating immunity, enhancing the body's antiviral ability, improving clinical symptoms, and reducing the toxic and side effects of antiviral drugs. AIDS is classified as either an internal or external cause or a combination of internal and external causes. The specific treatment adopts the method of nourishing qi and nourishing yin, strengthening the righteousness and eliminating pathogenic factors, and treating the symptom [8, 9]. Shenling Fuzheng capsules is a formula based on “Sijunzi Decoction”, including Radix Codonopsis, Ganoderma, Astragalus mongholicus, Atractylodes macrocephala, Black Ant, and Herba Gynostemmatis Pentaphylli, whose main function is to strengthen the spleen and benefit the qi. However, after stopping cART, the virus rebounds and is usually detected in plasma within a few weeks. Thus, viral load is the golden standard to evaluate the progression and prognosis effect of AIDS. Moreover, the expression level of the HIV-1 RNA gene can also reflect the activation status of HIV-1 virus. HIV-1 virus enters immune cells after infection, and its RNA is reverse transcribed into DNA and enters the nucleus. Most HIV-1 DNA is integrated into the human genome to form a stable viral reservoir (HIV-1DNA). HIV-1 DNA is used as a replication template to transcribe daughter RNA, translate proteins, and package them into daughter viruses. Under normal circumstances, the number and proportion of lymphocyte subsets in the normal human body are kept within a certain range to maintain the normal immune function of the body.

AIDS can impede or destroy immune function by targeting the primary immune cells, specifically CD4+ T cells and CD8+ T lymphocytes [10]. Some recent studies reported that the levels of CD4^+^/CD8^+^ T cells could better reflect the immune function of AIDS patients, compared to the expression of CD4^+^ T lymphocytes only [11, 12]. CD4 + T cells and CD8 + T cells are the main specific immune response cells in the body, which are closely related to the immune status of HIV-infected patients. Modern immunology suggests that HIV infection will lead to a decline in the function and number of CD4 cells in peripheral blood, resulting in the decline of immune function. CD4 cells are its main marker, and therefore, may serve as the main marker for immune evaluation of AIDS treatment [13, 14]. However, few studies have been carried out to reveal the relationship among the levels of CD4^+^/CD8^+^ T cells, the expression of the HIV-1 RNA pol gene, and viral load of AIDS patients after antiviral therapy.

Thus, to bridge this gap in the AIDS study, the present study attempted to compare the expression of the HIV-1 RNA pol gene, the levels of CD4^+^/CD8^+^ T cells, and viral load among 200 AIDS patients after antiviral treatment. The findings in this study are expected to provide more references for the antiviral therapy of AIDS.

## 2. Materials and Methods

### 2.1. Enrollment of the Subjects

A total of 200 AIDS patients that received antiviral treatment from January 2016 to January 2020 were selected as the research subjects. The original sample size calculation estimated that 200 patients in each group would be needed to detect a 3-point difference between groups in a 2-sided significance test with a power of 0.8 and an alpha error level of 0.05.

There were 106 males and 94 females, aged from 18 to 69 (42.59 ± 5.13) years. Permission and written informed consent were obtained from all the subjects and their relatives before commencement.

### 2.2. Inclusion and Exclusion Criteria

All patients were over 18 years old and were eligible for receiving antiviral treatment [15].

#### 2.2.1. Inclusion Criteria

1. Meet the above-mentioned HIV/AIDS diagnostic criteria, confirmed by the Center for Disease Control and Prevention of our hospital to be positive for HIV antibodies by Western Blot test, and issue a confirmation report
2. Age over 18
3. Those who meet the antivirus standards
4. Voluntarily signed the patient's informed consent, and can ensure regular follow-up and specimen collection

#### 2.2.2. Exclusion Criteria

1. Patients with severe hepatic and renal insufficiency, or concurrent severe cardiovascular and cerebrovascular, pulmonary and hematopoietic system, nervous system and other diseases
2. Patients with autoimmune diseases
3. Pregnant or breastfeeding women
4. Patients who have participated in clinical trials of other AIDS-related drugs within 1 year before the study drug treatment
5. Those who are allergic to the drugs taken by the institute during the experiment

### 2.3. Drugs, Treatment, and Test

All patients were treated under the HARRT regimen. Drugs used for the therapy included lamivudine (Guangshengtang, Fujian, H20113025), stavudine (Matrix, Xiamen, H20041726), nevirapine (Matrix, Xiamen, H20058461), and/or Efavirenz (Huahai, Zhejiang, H20133265).

The ratio of CD4^+^/CD8^+^ T cells in peripheral blood was determined. 3 mL of fasting venous blood of the patients were collected and transferred into an EDTA tube one day before the treatment or 3 months, 6 months, 12 months, and 24 months after the treatment. Subsequently, 0.5 mL of CD4^+^ antibody (BD Biosciences,565432, 1 : 1000) and CD8+ antibody (BD Biosciences, 5H10-1, 1 : 1000) was added, mixed gently, and incubated at 4°C for 30 minutes in the dark. The amounts of CD4^+^ and CD8^+^ T cells were analyzed by FACS (CountStar, Shanghai). The CD4^+^/CD8^+^ ratio was calculated.

For the determination of viral load, 3 mL of fasting venous blood was collected from the patients and transferred into an EDTA tube and then centrifuged for 30 minutes at 2000 r/min. Viral load was detected by quantitative Real-time PCR (RT-qPCR). RT-qPCR was performed using the ABI StepOne™ instrument. The reaction was set up in 20 *μ*L containing 10 *μ*L of RealQ Plus Master mix for Probe (Amplicon, Denmark), 0.4 *μ*M of each HIV primer, 0.2 *μ*M of each internal control (IC) primer, 0.25 *μ*M HIV probe, 0.125 *μ*M IC probes, and 5 *μ*l of cDNA. The amplification profile consisted of a single cycle of enzyme activation at 95°C for 15 min followed by 45 cycles of denaturation at 95°C for 10 s, annealing at 54°C for 30 s, and 72°C for 30 s with a single fluorescence acquisition at channel FAM/HEX. A nontemplate control was included in each qPCR assay. All the procedure was performed according to MIQE guidelines [16, 17].

For the HIV-1 RNA pol gene expression, 5 mL of fasting venous blood was collected from the patients and transferred into an anticoagulant tube, and centrifuged through the Ficoll gradient for the isolation of monocytes. Specifically, 5 mL of peripheral blood were added into 0.6 mL of heparin and mixed with an equal volume of Hank's solution. Ficoll was carefully overlaid with blood in a new tube and centrifuged at 1500 r/min for 10 min. After centrifugation, an opaque band that contained monocytes at the interface between blood and Ficoll was collected and transferred into another tube. Thereafter, the band was mixed with an equal volume of the Hank's solution and centrifuged at 1000 r/min for 10 min. After centrifugation, the supernatant was removed and the cell pellets were washed twice with an equal volume of the Hank's solution. Finally, the cell pellets were re-suspended in 1 mL of RPMI-1640 culture medium and stored at 4°C for future use. The nested polymerase chain reaction (nPCR) was used to detect the HIV-1 RNA pol gene expression. The PCR reaction volume for both outside HIV-1 DNA primer and inner HIV-1 DNA primer was 25 PL. The amplification parameters of the outside HIV-1 primer were the same as that of the inner HIV-1 primer. The former was carried out for a total of 43 cycles, in contrast to 35 cycles for the latter. The positive and negative controls were set up for PCR amplification to obviate the false positive or negative results of PCR amplification.

Biochemical indicators (alanine aminotransferase (ALT), white blood cell (WBC) count, Serum creatinine (Cr), total cholesterol (TC), triglyceride (TG), and platelet (PLT), aspartate aminotransferase (AST), red blood cell (RBC), and neutrophil (NEU)) in the venous blood collected 1 day before the treatment or 24 months after the treatment was also determined by an automatic biochemical analyzer (Beckman Coulter).

The patients in both groups received 148 mg of Shenling Fuzheng capsules (37 g/capsule) thrice daily.

### 2.4. Observant Indexes

For all the 200 participants in the present study, the observant indexes included (1) the expression level of the HIV-1 RNA pol gene before and after treatment; (2) the viral load before and after treatment; (3) peripheral blood CD+3, CD4+, and CD+8 cell counts (pcs/*μ*l) were measured at enrollment and at the completion of treatment using a FACS Calibur flow cytometer from BD, USA. One follow-up test was performed 6 months after treatment. Detection of CD+3, CD4+, CD+8 cell percentage and CD4+/CD+8 in peripheral blood was performed using BECKMAN Cytomics FC500 Flow Cytometry Analyzer and BFCKMAN COULTER reagents from USA; (4) the correlation between the HIV-1 RNA gene and the viral load using logstic regression analysis; and (5) ALT, WBC, Cr, TC, TG, PLT, AST, RBC and NEU% before and after treatment.

### 2.5. Ethics

Before enrollment, the study obtained the informed consent of the patients. This study protocol was approved by the Ethics Committee of Baoding People's Hospital, Ethics number: 2019-03. It was confirmed that informed consent for our experiments had been obtained from all patients. All procedures complied with the ethical guidelines of the Declaration of Helsinki.

### 2.6. Statistical Analysis

Statistical analysis was performed with SPSS software version 25.0 and quantitative data were presented as mean ± standard deviation (SD). The transformed data were tested for normality using Shapiro-Wilk, and all log-transformed variables were normally distributed. The Mann–Whitney *U* test was used for the intergroup analysis. Enumeration data were presented as percentage (%) and comparisons between two groups were analyzed by the Chi-squared Test. Logstic regression analysis was used to study the correlations of relevant indexes. Differences between samples were examined using paired two-sided Student's *t*-test. If the *p* value is less than 0.05, it means that there is a statistically significant difference. The Gradpad Prism version 7.0 was used for generation of graphs.

## 3. Results

### 3.1. The Levels of the HIV-1 RNA Pol Gene Expression, CD4^+^/CD8^+^ T Cells, and Viral Load

The HIV-1 RNA expression levels were significantly reduced following 3-month, 6-month, and 12-month antiviral treatment, suggesting that antiviral treatment might effectively limit the HIV-1 RNA pol gene expression in AIDS patients (*P* < 0.001) (Figure 1(a)).

The peripheral CD4+/CD8+ T cell levels of 200 patients elevated considerably after therapy, suggesting that antiviral medication could successfully activate the immune system and boost AIDS patients' immunity (*P* < 0.001, Figure 1(b)).

The viral load of 200 individuals decreased dramatically following treatment, indicating that antiviral therapy may successfully manage the quantity of HIV virus (*P* < 0.001, Figure 1(c)).

### 3.2. Correlation between Viral Load and the HIV-1 RNA Gene Expression or CD4^+^/CD8^+^T Cells

After 24 months of therapy, a logistic analysis was undertaken to further examine the association between viral load and HIV-1 RNA gene expression or CD4+/CD8+ T cells. Patients' viral loads were positively connected with HIV-1 RNA and negatively correlated with CD4+/CD8+ (*P* < 0.01, Figure 2).

### 3.3. Biochemical Indicators

After 24 months' treatment, levels of ALT, WBC, Cr, TC, TG, and PLT significantly increased (ALT: *P* = 0.0086; WBC: *P* = 0.0012; Cr: *P* = 0.0058; TC: *P* = 0.0072; TG: 0.0049; PLT: *P* = 0.0069, Figure 3), whereas levels of AST, RBC, and NEU% showed no marked changes (AST: *P* = 0.0523; RBC: *P* = 0.0934; NEU%: *P* = 0.9999). Thus, antiviral therapy may be harmful to AIDS patients' hepatic and renal functioning, as well as lower plasma lipid levels.

## 4. Discussion

AIDS was first discovered in the early 1980s and has an extremely high fatality rate. After the pathogen invades the human body, it directly parasitizes the target cells of the host. After a long period of latency, the human immune system and its function are compromised, and it eventually develops into AIDS and endangers the patient's life. After more than 20 years of research by the international medical community, more evidence about its pathogens and pathological changes have been identified, but clinical treatment is still lagging behind [18, 19]. AIDS is spread through sexual, blood, or maternal-infant manner [20, 21]. It causes severe adverse impact on immune function of patients and results in multiple immune diseases [22]. HARRT therapy is a well-developed treatment for AIDS, with multiple merits including inhibition of the duplication and propagation of HIV virus, enhancement of the immune function of patients, reduction of the risk of complications, and increase in the survival rate of patients [23, 24]. HAART, also known as “cocktail therapy”, was first proposed by Chinese-American scientist Dr. He Dayi and French scientist Prof. Autran in the 1990s. It has been verified that high-efficiency antiretroviral therapy inhibits virus replication, promotes immune reconstruction to a certain extent, and finally restores various immune abnormalities caused by HIV infection [25].

According to the knowledge of many physicians since its discovery, AIDS can be categorized into plague, epidemic virus, cold temperature, and accumulation of strain in TCM. From the perspective of TCM syndrome differentiation, the etiology of AIDS is related to the pathogenesis of exogenous damp-heat epidemic, and its nature is mainly damp-heat. The key factor of pathogenicity lies in the weakness of the righteous qi in the human body, and the pathogenic qi of the epidemic takes advantage of the deficiency, with the disease located in the liver, spleen, and kidney [26]. From the perspective of the entire etiology of AIDS, it is caused by poisonous pathogens that invade the body. When the poison enters the body, it breeds various poisonous evils, such as damp-heat poison, and cold-damp poison. Endogenous poisonous evils are usually formed by the mutual accumulation of pathological products such as phlegm, water, congestion, and exogenous evils. Damp poisons always run through the entire process of the occurrence, development and evolution of AIDS, plus the unique pathogenic characteristics and evolution of AIDS, resulting in the further development of the disease [27, 28].

The main drug composition of Shenling Fuzheng capsules are Codonopsis, Astragalus, Poria, Atractylodes, Gynostemma, Black Ant, Ganoderma Lucidum, and Fufang Teng. Functions and indications are invigorating the spleen and removing dampness and nourishing qi and blood. Modern pharmacological studies have shown that Codonopsis has the functions of regulating human immune function, promoting hematopoietic function, antioxidation, and antifatigue. Radix Codonopsis is involved in bidirectional immunomodulatory effects, and Ganoderma induces the production and activation of macrophage and NK cell activities in humans. Among them, Codonopsis polysaccharide can significantly increase the content of IgG and IgM in the serum of the mouse model, thereby improving the immune function of the body. Codonopsis polysaccharide can stimulate the proliferation of lymphocytes and improve the body's cellular immunity. Astragalus has the effect of enhancing the body's humoral immunity. Injection of a certain amount of astragalus injection into the immunocompromised mice improves the humoral immune response of goat erythrocytes in vivo, and its active ingredients can increase the level of specific antibodies in the body, suggesting that Shenling Fuzheng capsule can enhance the body's immunity to resist external pathogens [29–31].

The level of the HIV-1 RNA pol gene expression can represent the active state of HIV virus in AIDS patients [32]. The present study used nPCR to detect the HIV-1 RNA pol expression of AIDS patients before and after treatment, and found that after treatment, the HIV-1 RNA pol expression significantly reduced, indicating that the HIV gene expression was remarkably suppressed after treatment. Moreover, the viral load, the number of virus per milliliter of blood, is also another important marker to evaluate the therapeutic efficacy [33]. Here, 200 patients in the present study were detected to have significant reduction of viral load after treatment, proving that antiviral treatment takes effect. The reason may be that HAART reduces the drug resistance caused by a single drug, inhibits the replication of the virus to the greatest extent, and restores part or all of the damaged immune function, thereby delaying the progression of the disease, prolonging the life of the patient, and improving the quality of life. The therapy combines protease inhibitors with a variety of antiviral drugs to effectively control AIDS. In addition, TCM has a variety of biological activities, which may play a certain role in inhibiting the apoptosis of HIV/AIDS patients. It can improve the medication compliance of HIV/AIDS patients and reduce the drug resistance of HAART and its side effects. The method of the current study inhibited the apoptosis of CD4+ T lymphocytes, so as to prolong the lifespan of normal CD4+ cells and HIV-infected cells, and maintain the number of CD4+ cells in the body at a relatively stable level [34, 35].

The correlation between CD4^+^/CD8^+^ T cell and the status of immune function of AIDS patients was widely validated [36, 37]. It has been discovered that early and continuous treatment of AIDS patients is critical for improving their CD4^+^/CD8^+^ T cell level [38]. A CD4+/CD8+ T ratio greater than one was reported in only 20% of patients in their research, suggesting that early therapy and maintenance of treatment compliance in AIDS patients are critical to enhance the CD4+/CD8+ ratio and maximize immunological reconstitution. Furthermore, it has been found that CD4+, CD8+, and CD4+/CD8+ ratios were considerably lower in AIDS patients than in healthy populations [39]. Compared to CD4^+^ and CD8^+^, the CD4^+^/CD8^+^ ratio is a more specific and sensitive indicator in AIDS diagnosis. In this research, after antiviral treatment of 200 patients, their CD4^+^/CD8^+^ ratio increased significantly, suggesting that the humoral immunity of the patients was activated, which positively contributed to the resistance to opportunistic infections, thus improving the function of human organ systems and facilitating the recovery of the patients. It is worthwhile to further investigate at the cellular molecular level that Shenling Fuzheng capsule promotes the recovery of CD4+ T cells in patients with poor immune reconstitution.

The present research also investigated the correlation between HIV-1 RNA and viral load or CD4^+^/CD8^+^ ratio. Results showed that HIV-1 RNA was positively related to viral load, while negatively related with CD4^+^/CD8^+^ ratio. HIV-1 RNA and viral load expression levels can indicate the active state of HIV-1 virus in AIDS patients [40, 41]. Other observations showed that after various interventions of AIDS patients, their HIV-1 RNA expression level and viral load were drastically altered [42], and HIV-1 RNA and viral load can be used to evaluate the prognosis effect of AIDS patients. Another study found that HIV infection can lead to significant reduction of CD4^+^/CD8^+^ ratio [43]. The reduction of CD4^+^/CD8^+^ ratio indicated that the immune function was markedly decreased, which promotes the further increase of HIV-1 RNA expression, indicating an interplay between HIV-1 RNA and CD4^+^/CD8^+^.

With the progression of disease and growth of age, long-term medication is associated with multiple complications such as hepatic and rental dysfunction, and cardiovascular diseases in AIDS patients [44, 45]. As a result, several biochemical indications before and after AIDS treatment were compared. The results showed that ALT, WBC, Cr, TC, TG, and PLT levels were all considerably increased. Long-term use of antiviral medications such as lamivudine, stavudine, and nevirapine, will undermine the hepatic and rental function to varying degrees, resulting in aberrant biochemical indices such as ALT [46]. Increased TC and TG can induce cardiovascular diseases [47]. Therefore, during the medication of AIDS patients, regular examination of hepatic and rental function and cardiovascular status should be done to avoid other complications. Increased PLT level after treatment might be attributed to decreased HIV virus in megakaryocyte after medication and restored the clump of platelets [48]. WBC elevation might come from the improvement of blood circulation and blood cell quality after antiviral administration, which might reduce the occurrence of complications of AIDS patients [49, 50]. Further research is warranted by grouping the patients according to clinical therapeutic efficacy to compare the HIV-1 pol gene expression and peripheral CD4^+^/CD8^+^ T cell levels under different therapeutic effects.

Compared with conventional tonics, the Shenling Fuzheng capsules in the present study are portable and efficacious, which provides some evidence-based basis for the treatment of AIDs with traditional Chinese medicine. In addition, differing from conventional clinical observational studies, the present study also observed the expression of the HIV-1 pol gene and analyzed the effect of drugs on the gene from a genetic perspective. This provides ideas for future clinicians for diagnosis and treatment and also provides a reference value for future drug design based on the HIV-1 pol gene. There are still some limitations in this study. These are the following: (1) This experiment is a short-term observational study of the curative effect, which cannot systematically observe the long-term clinical outcomes, and the relatively small sample size and short observation period of this study will bias the study results. (2) Due to the overall high level of CD4+ T lymphocyte counts in HIA/AIDS patients enrolled in this trial, and there are many types of HAART regimens, the enrolled HIV/AIDS patients failed to maintain consistent treatment regimens. This may be one of the factors compromising the test results. Therefore, in the subsequent research, the consistency of the experimental conditions between the groups should be maintained as much as possible, and the factors that may affect the experimental results should be excluded.

## 5. Conclusion

HIV-1 RNA pol gene expression and viral load in AIDS patients decreased considerably after antiviral treatment, but peripheral CD4+/CD8+ T cells rose dramatically. The present study showed that antiviral medications effectively reduce HIV-1 RNA POL gene expression and viral load in AIDS patients while increasing the expression level of CD4+/CD8+ T cells in peripheral blood. Furthermore, the sensitivity and specificity of relevant indicators may be used to assess the prognostic impacts of AIDS patients.

A large number of clinical trials have confirmed that TCM combined with HAART can alleviate the symptoms, improve the quality of survival and enhance the immune function of HIV patients. However, there is no standardized understanding of the etiology and pathogenesis of HIV in TCM, and the mechanism of action of TCM used for the treatment of HIV remains unknown. The benefits of holistic, diverse, and multitargeted TCM treatment still require further investigation.

## Figures and Tables

**Figure 1:** Comparison of therapeutic effects before and after antiviral treatment. (a) Comparison of HIV-1 RNA pol gene expression of 200 patients before and after treatment, ^∗∗^*P* < 0.001. Antiviral treatment might effectively limit the HIV-1 RNA pol gene expression in AIDS patients. (b) Comparison of peripheral CD4^+^/CD8^+^ T cell of 200 patients before and after treatment, ^∗∗^*P* < 0.001 Antiviral medication can successfully activate the immune system and boost AIDS patients' immunity. (c) Comparison of viral load of 200 patients before and after treatment, ^∗∗^*P* < 0.001. Antiviral therapy may successfully manage the quantity of HIV virus.

**Figure 2:** Correlation analysis between viral load and HIV-1 RNA or CD4^+^/CD8^+^. (a) Viral load was positively related with HIV-1 RNA, *r* = 0.634, *P* = 0.006. (b) Viral load was negatively related with CD4^+^/CD8^+^, *r* = −0.652, *P* = 0.003.

**Figure 3:** Biochemical indicators of 200 patients before and after antiviral treatment. (a) ALT; (b) AST; (c) WBC; (d) Cr; (e) RBC; (f) NEU; (g) TC; (h) TG; (i) PLT; ^∗∗^*P* < 0.001. Antiviral medication may impair hepatic and renal function in AIDS patients, as well as reduce plasma lipid levels.

## Data Availability

All data generated or analyzed during this study are included in this published article.
